# Lymph Node Metastases Detection Using Gd_2_O_3_@PCD as Novel Multifunctional Contrast Imaging Agent in Metabolic Magnetic Resonance Molecular Imaging

**DOI:** 10.1155/2022/5425851

**Published:** 2022-10-12

**Authors:** Z. Rasouli, N. Riyahi-Alam, M. Khoobi, S. Haghgoo, E. Gholibegloo, A. Ebrahimpour, Ashouri H, H. Hashemi

**Affiliations:** ^1^Medical Physics & Biomedical Engineering Department, School of Medicine, Tehran University of Medical Sciences (TUMS), Tehran, Iran; ^2^Medical Imaging Center, Motahari Hospital, Jahrom University of Medical Sciences (JUMS), Jahrom, Iran; ^3^Concordia University, Perform Center, Montreal, Quebec, Canada; ^4^Biomaterials Group, The Institute of Pharmaceutical Sciences (TIPS), Tehran University of Medical Sciences, Tehran, Iran; ^5^Department of Medicinal Chemistry, Faculty of Pharmacy, Tehran University of Medical Sciences, Tehran, Iran; ^6^Pharmaceutical Department, Food and Drug Laboratory Research Center, Ministry of Health, Tehran, Iran; ^7^Department of Radiopharmacy, Faculty of Pharmacy, Tehran University of Medical Sciences, Tehran, Iran; ^8^Medical Imaging Center of Imam Complex Hospital, Tehran University of Medical Sciences (TUMS), Tehran, Iran; ^9^Department of Radiology, School of Medicine, Tehran University of Medical Sciences (TUMS), Tehran, Iran

## Abstract

Axillary lymph node detection is crucial to staging and prognosis of the lymph node metastatic spread in breast cancer. Currently, lymphoscintigraphy and blue dye, as the conventional methods to localize sentinel lymph nodes (SLNs), are invasive and can only be performed during surgery. This study has had a novel hybrid gadolinium oxide nanoparticle coating with Cyclodextrin-based polyester as a high-relaxivity T_1_ magnetic resonance molecular imaging (MRMI) contrast agent (CA). Twelve female BALB/c mice were randomly divided into three groups of four mice; each group was injected with 4T_1_ cells to obtain metastasis lymph nodes and diagnosed by using the 3D T_1_W (VIBE) MRI (Siemens 3T, Prisma). The synthesized Gd_2_O_3_@PCD nanoparticles with a suitable particle size range of 20–40 nm have had much higher longitudinal relaxivity (*r*_1_) for Gd_2_O_3_@PCD and Gd-DOTA (Dotarem) with the values of 3.98 mM^−1^·s^−1^ ± 0.003 and 2.71 mM^−1^·s^−1^ ± 0.005, respectively. Identical MR images in coronal views were subsequently obtained to create time-intensity curves of the right axillary lymph nodes and to measure the contrast ratio (CR). The peak CR and qualitative assessment of axillary lymph nodes at five-time points were evaluated. After subcutaneous injection, the contrast ratio of axillary lymph node and tumor in mice exhibited CR peak of Gd_2_O_3_@PCD and Dotarem with the values of 2.21 ± 0.06 and 0.40 ± 0.004 for lymph node and 2.54 ± 0.04 and 1.21 ± 0.007 for the tumor, respectively. Furthermore, the lumbar-aortic lymph node is weakly visible in the original coronal image. In conclusion, the use of Gd_2_O_3_@PCD nanoparticles as novel MRMI CAs enables high resolution for the detection of lymph node metastasis in mice with the potential capability for breast cancer diagnostic imaging.

## 1. Introduction

Breast cancer is the most common cancer diagnosed worldwide, with more than 2 million cases in 2020 [1]. The presence of lymph node (LN) metastases that lead to malignancy breast cancer spread to axillary sentinel lymph nodes (ASLNs) is one of the most important predictors of patient survival but with major prognostic implications and management [2, 3]. Typically, breast cancer metastasizes to the ASLN and considered the first node to drain the tumor's lymphatic fluid [4, 5]. Therefore, the detection of ASLN metastases is crucial to staging and prognosis.

Currently, lymphoscintigraphy as the most widely used method to localize sentinel lymph node (SLN), has some diagnostic and implementation disadvantages of associated precautions by using a radioactive tracer, while the poor image quality and low spatial resolution of scintigrams cannot provide anatomical details, as well [6, 7]. Intraoperative lymph node imaging with the administration of Isosulfan blue (blue dye) is another commonly used technique to identify SLN, but it is invasive and can only be performed during surgery [8].

MRI techniques facilitate the quantification of anatomical changes related to the development of pathologic states, leading to the early diagnosis of diseases such as cancer [9]. In magnetic resonance molecular imaging (MRMI), contrast agents (CAs) are necessary to achieve a high spatial resolution in studies of the lymphatic system, required to develop a new lymphographic CA [10]. Lymphangiography using MRI (MRL) is a relatively new procedure consisting of the acquisition of MRI after interstitial injection of CAs. MRL with gadolinium-based CA (Gd-MRL) can generate high spatial resolution images of lymph nodes [11–16]. Interstitial administration of CA enables assessing the lymphatic system with lower doses and allows morphological and functional evaluations of the lymphatic system to detect SLN [17, 18]. This method can be used for the detection of SLN in the drainage from a tumor site and indicate early metastases [10]. For the interstitial MRL, several T_1_ agents and extracellular agents such as gadopentetate dimeglumine can be used for MRL, even though they have demonstrated nonspecific distribution, rapid elimination, and effect on nephrogenic systemic fibrosis (NSF) [19–21].

In recent years, several different CA, as well as nanomaterials, have also been developed and tested in MRMI for imaging of the lymphatic system using interstitial injection, whereby the CAs absorbed and transported from the interstitial tissue into the collector lymphatics [22–28]. Compared to conventional CAs, nanoparticles (NP) CAs offer several merits that one of them being loadability, in which the concentration of the CA can be adjusted to suit the particular NP in the synthesis process. A major advantage of using nanoparticles as CAs is their ability to target specific areas. Paramagnetic nanoparticles can be used in targeted imaging, cell tracking, and multimodal imaging. [13, 29–34].

Targeted CAs with MRI enables noninvasive detection and characterization of biological changes at the molecular level. CAs can target specific receptors, molecules, or cell types passively or actively by binding selectively to molecular targets due to their distribution characteristics that favor specific tissues or cell types. *β*-Cyclodextrin (*β* CD) ring, containing seven glucose monomers, is a coating agent widely used for inorganic nanoparticle modification because of its biocompatibility, amphiphilicity, and host-guest interactions [9, 10, 35]. Targeted CAs, Gd_2_O_3_@Polycyclodextrin, were evaluated for malignant lymph nodes based on the difference in glucose utilization between the tumor and normal tissue for interstitial MRL in mouse models compared to a conventional CA, Gd-DOTA (Dotarem). Previous studies have been undertaken to improve the water solubility of the Gd CA by introducing various groups of sugar into their structures [36, 37]. In this study, to overcome the abovementioned problems, variations of NPs with CD used in this study, a type of macrocyclic oligosaccharide, have been utilized in several ways due to favorable properties such as truncated cone chemical structure with outstanding biodegradability [37].

## 2. Materials and Methods

### 2.1. Characterization

Analyses of the hydrodynamic size distribution (DLS) and zeta potential were performed in deionized water at room temperature by using a zeta sizer (ZEN3600, Malvern), and the morphology of the dried samples was determined by using transmission electron microscopy, TEM (CM30, Philips) operating at 60 kV.

### 2.2. Relaxivity Measurement

After synthesis and characterization of PCD coated Gd_2_O_3_ (Gd_2_O_3_@PCD) based on our previous research [37–39], for longitudinal relaxivity (*r*_1_) evaluation, Gd_2_O_3_@PCD NPs were dispersed in water with various Gd concentrations (0, 0.04, 0.08, 0.16, 0.32, 0.64, and 1.28 mM). Dotarem was prepared using the same concentration of Gd^+3^ as the control sample, and all samples were dispersed in a 2% agarose (Sigma-Aldrich) solution. Longitudinal relaxivity was measured using an MRI unit (Siemens 3 T, Prisma) with a head coil. T_1_ -weighted (W) images were obtained with a conventional spin-echo sequence that contained these parameters: TR/TE = 50, 200, 400, 600, 800, 1100, 1300, 1500, 1800, and 2000/15 ms, slice thickness = 4 mm, flip angle: 90°, number of signal averages of 3, and 128 by 128 mm^2^ field of view. Signal intensities were obtained with manually drawn regions of interest (ROI) for each sample. Relaxation rates, *R*_1_ (1/T_1_), were calculated by MATLAB software.

### 2.3. Mouse Tumor Model

A total of 14 female BALB/c mice (5 weeks old) were obtained from the Pasteur Institute in Iran. Animal experiments were carried out according to the European Community Guidelines, an accepted set of guidelines for the use of laboratory animals, with approval from the local ethics committee of Teheran University of Medical Sciences (TUMS), Tehran, Iran. The animal tumor model was established on 4 to 5-week-old BALB/c mice (25 g) by subcutaneously inoculating 4T_1_ cell lines (epithelial breast carcinoma cell lines). MR imaging (Siemens 3 T, Prisma) was carried out after 21 to 23 days after tumor inoculation when the tumor size reached 1.0–2.0 cm. The mice were randomly divided into three groups (*n* = 4 mice/group). The mice were randomly divided into three groups: two experimental groups (*n* = 8) and one control group (*n* = 4). In the experimental group, mice were injected with 10 *μ*L of 0.6 mM Dotarem or Gd NPs. One group of mice was injected with saline (PBS) as a control.

Following necropsy, two random mice were dissected to assess body weight and tumor metastasis to lymph nodes. In order to, the mouse was sacrificed using an isoflurane anesthetic, the skin of the posterior limb was removed, and SLNs were photographed by using a Canon digital camera. The animals were euthanized, and the harvested tissues' tumor mass and lymph node were fixed in the 10% neutral buffered formalin (NBF, PH. 7.26) for 48 h and then processed and embedded in paraffin. The 5 *µ*m thick sections were prepared and stained with hematoxylin and eosin (H&E). The histological slides were assessed by the independent reviewer by using light microscopy (Olympus, Japan).

### 2.4. In Vivo MR Imaging

All experiments using mice (*n* = 12) were performed by the Iran National Institutes of Health guidelines for the care and use of laboratory research animals. MRI (Siemens 3 T, Prisma) was repeated three times in three mice groups for each CAs. Animals were anesthetized with 3% isoflurane by using an MR-compatible mobile inhalation system (DRE Inc, Louisville, KY) and sedated with 2.5% isoflurane during imaging. Animals were placed prone on a custom platform in the RF coil, with legs loosely taped to a water-filled 15 ml test tube at the same level to maintain positioning and to optimize magnetic field homogeneity. 10 *μ*L of 0.6 mM Gd_2_O_3_@PCD NPs were subcutaneously injected into the mice's right hind paw, and then MRI was performed (Figure 1).

An optimized MR protocol was developed to provide adequate signal-to-noise and scan time paired with high spatial resolution. Imaging was performed by using a coronal T_1_-weighted 3D fast gradient echo sequence, with TR/TE: 6 msec/3 msec; flip angle: 12°; field of view: 44 × 44 mm; imaging matrix: 316 × 243; slice thickness: 2 mm. A precontrast acquisition (*t* = 0 min) was acquired, followed by sequential postcontrast acquisitions at 15, 30, 45, 60, and 120 min. For each CAs, a T_1_-W image was taken. To prevent confounding partial volume effects at the corners of the lymph nodes, the top and bottom slices were not included in the data analysis. To measure the signal intensities, a polygonal ROI was set up around the tumor and ASLN.

Then the contrast ratio (CR) at each time point was calculated using the following equation:

(1) $$\begin{array}{c} CR=\frac{\left(SI_{after}-SI_{before}\right)}{SI_{before}}, \end{array}$$

where *SI*_*after*_ represents the after-contrast normalized lymph node signal intensity and *SI*_*before*_ represents the before-contrast normalized lymph node signal intensity.

In the metastasised lymph node mouse model, we analyzed quantitatively the time course of contrast enhancement in the right lymph nodes that were markedly enlarged in all mice. By measuring the signal intensities, ROIs for each lymph node image in mice were also evaluated by two radiologists using Siemens Leonardo image workstations without knowing the other's radiologic evaluation results on blind or two blind analyses. Results of all tests were expressed as mean differences, and significance was determined by a *t*-test. *P* < 0.05 indicated a statistically significant difference.

## 3. Results

TEM images revealed spherical and uniform NPs and were visualized separately with clear grains in nano-dimensions in the range of 20–30 nm (Figure 2(a)). The size and Poly Disparity index (PDI) by DLS showed that Gd_2_O_3_ nanoparticles had a hydrodynamic diameter distribution of 45 ± 7.6 nm with a PDI of 0.36. Despite their different sizes, PDIs of the NPs showed acceptable ranges of less than 0.5. The Zeta potentials value of Gd_2_O_3_ and Gd_2_O_3_@PCD NPs were (+17.5 mv) and (-37.5 mv), respectively, which confirm Gd_2_O_3_ coating with PCD (Figures 2(b) and 2(c)).

### 3.1. Relaxivity Measurement

The Gd_2_O_3_@ PCD NPs were found to efficiently shorten the T_1_ and significantly increase signal intensity in T_1_-weighted images compared to Dotarem, with low concentrations of could be detected with MRI (Figures 3(a) and 3(b)). The degree of contrast enhancement in T_1_W images for all groups was found to be directly related to the concentration of Gd ions. For the quantitative evaluation, *r*_1_ relaxivities of the particles were calculated by measuring the relaxation rate as a function of Gd ion concentration. The longitudinal relaxivity of the Gd_2_O_3_@ PCD was found to be 3.98 mM^−1^·s^−1^ vs. 2.71 mM^−1^·s^−1^ for Dotarem (Figure 3).

After mice were dissected, we examined the LNs under the microscope to identify metastatic tumor processes that included metastases in the SLN, blood vessels, and lymphatic vessels. Focal metastasis of breast cancer (black arrows in Figure 4) was seen in the harvested lymph node. Many disproportionate tumor cells (anisocytosis), nuclear polymorphism (anisokaryosis, +3), and prominent nucleoli were seen in tumor mass sections (Figure 4).

### 3.2. In Vivo Lymph Node Imaging

The study compared Dotarem with Gd_2_O_3_ @ PCD nanoparticles for the detection of SLN in tumoral mice. CAs were injected subcutaneously into the right hint paw and drained into the right SLN (Figure 5(a)). Following injection with Gd_2_O_3_@PCD NPs, a series of images was obtained after 15, 30, 45, 60, and 120 minutes. Contrast enhancement of axillary lymph node and tumor in mice exhibited CR peak of Gd_2_O_3_@PCD and Dotarem with the values of 2.21 and 0.40 for lymph node and 2.54 and 1.21 for the tumor, respectively. Dotarem uptake into the tumor margins and SLN was detected weakly, respectively, 15 and 45 min after injection (Figures 5–8).

The Dotarem integrated density changed similarly between precontrast and 15, 30, 45, and 120 minutes postcontrast for the ALN. Gd_2_O_3_@PCD showed a strong increase in contrast uptake in the ALN at 30 min (Figure 6). 45 minutes postcontrast, the lymph nodes showed decreased contrast levels, which is probably due to lymphatic drainage to more SLN at this time. Only Gd_2_O_3_@PCD had significantly greater CA uptake in tumor-draining ALN and lumbar lymph nodes. Figures 6 and 7(b) show that Dotarem has similar CA uptake in the lymph node region. As a result, Gd_2_O_3_@PCD was the only CA able to demonstrate tumor-induced CA uptake at *t* = 15 minutes and continued higher CA accumulation within the ALN at *t* = 30 minutes.

## 4. Discussion

In many cancers, especially breast cancer, staging is affected by lymph node status. Although tissue characterization by histopathology of biopsy samples may improve staging, noninvasive staging is more acceptable both to patients and clinicians. Several imaging techniques can facilitate this process. Noninvasive techniques such as computed tomography and MRI detect lymph node abnormality by nodal enlargement, but this does not always imply malignancy. On the other hand, some nodes are infiltrated or replaced with tumors without changing in size. The methods have this serious problem. Due to this, a great deal of attention has been directed toward developing CA and radio-labelled complexes for better cancer detection and characterization of individual lymph node tumors [40]. Detection of early metastases within the SLN requires a high target to the background. By targeting nanoparticles, we have increased tumor specificity compared to normal organs to a moderate degree. To promote NP accumulation at the site of interest, active or passive targeting is the ideal solution [41]. Although Gd-based nanoparticles CAs MRL could verify the lymph node imaging, SLNs imaging with MRI has been accompanied by issues, such as no specificity, short durations, and high doses of CAs, which may be associated with long-term toxicities [19–21]. CAs for MRMI may allow SLN imaging to be performed in vivo without these disadvantages.

The molecular size of the CA can significantly influence lymph node imaging, while the optimum size, which preferably flows through the lymphatic system, is unclear. A good agent for identifying SLNs would be administered in high concentration to the lymph nodes for imaging, with a low background concentration in the surrounding normal tissues [42]. SLN imaging requires a nanoprobe whose properties correlate with its shape, size, function, and biocompatibility. Researchers have utilized a variety of nanomaterials in vivo to investigate the lymphatics by using interstitial injections, whereby the CAs are absorbed from the interstitial tissue and transported to the collector lymphatics [25, 26, 28]. Therefore, a method of enhancing the lymphatic structures is also necessary to achieve sufficient SNR. Recently, superparamagnetic iron oxide NPs (SPION)-MR lymphography and iopamidol-CT lymphography with interstitial injection of CAs for breast cancer has been reported. Compared with SPION-MRL, Gd-MRL is more economical and convenient, since SPIONs beside as a negative CAs is difficult to image the lymphatic vessels due to blossom artifact among the dark background, and compared with iopamidol-CT lymphography, Gd-MRL lacks radiation exposure, the less possibility of anaphylactic shock, and nephrotoxic impairment, as well [19, 20, 28, 29]. The Morawitz studies have shown that PET/MRI is more accurate than MRI and CT for diagnosing lymph node metastasis in patients with primary breast cancer and for nodal staging [43]. We propose to compare it with MRMI, which uses a targeted and noninvasive CA. The use of a CA helps identify the SLN, and a high-resolution MRI provides accurate information about the location and properties of the node. Overall, these MRI contrast agents provide a framework for achieving a greater level of accuracy from MRI as a low-cost, more accessible facility, nonradioactive source of radiation, and highly sensitive facility to propose as an alternative to PET nuclear medicine.

To overcome the problems of morphological SLN detection in conventional MR lymphangiography methods, in this group, previous studies have been undertaken to improve the structural and metabolically CA providing water solubility of the Gd CA by introducing various groups of sugar (Gd-DEG-DG, Gd DTPA-DG) into their chemical structures [32, 38, 39]. In other research by this group, variations of NPs with CD and *β*CD as a coating agent for inorganic NP modification also have been utilized in several ways due to favorable properties such as truncated cone chemical structure with outstanding biocompatibility and biodegradability [37]. For this purpose, instead of conventional structural covering (DTPA, DOTA, DOPTA, DTPA-BMA), Gd condensation polymerization was carried out between CD and DTPA-DA in the presence of Gd_2_O_3_ NPs. Resulting in CD-based polyester containing appropriate functional groups for chelating of Gd_2_O_3_ core and further functionalization. The passive targeting capability of Gd_2_O_3_@PCD nanoparticles allows them to accumulate in metastatic lymph nodes rather than blood vessels, which makes them highly selective.

Nanoparticle characteristics, particle size, and surface charge are widely known to affect the uptake pathway and effectiveness of molecules in cells. In this study, the positive charge of the naked Gd_2_O_3_ NPs reduced to negative, which is due to the negative charge of the polymer layer on the surface of the NPs after coating, resulting from hydroxyl and carboxyl groups of the polymer. As well, the achieved molecular size of the CA could significantly influence lymph node imaging with the proper size of 20–40 nm, which preferably flows them through the lymphatic system. In this regard, Gd_2_O_3_@PCD NPs were found to efficiently shorten the T_1_ leading to a significant increase in the signal intensity in T_1_W images compared to Dotarem (Figures 2 and 3). Considering the *r*_1_ values of 3.98 vs. 2.71 mM^−1^·S^−1^ for Gd_2_O_3_@PCD and Dotarem, respectively, the low concentrations of these nanoparticles can be detected with MRI, showing the proper concentration in the range of 0.04–1.2 mM of this new CA in-vitro imaging. This result is consistent with the previous study's claim that Gd chelates in nanoscale carriers improve MRI relaxivity [24, 37, 39, 44, 45]. Consistently, the improved MRI relaxivity is related to the smaller nanoscale particle diameter. The lower dose concentration needed to achieve visual effect in this study was desirable because reducing the dose of MRI CAs based on Gd ions can circumvent long-term toxic effects, such as chronic kidney disease.

In addition, according to toxicology results, Gd_2_O_3_ coating by PCD led to a reduction of Gd leakage. Cell viability for normal human breast cell line (MCF-10A) showed no obvious decrease in cell viability observed with various concentrations of Gd_2_O_3_@PCD NPs (up to 50 *μ*g/mL) for 24 h incubation time. As a result of their selective toxicity and higher relaxivity than commercial Dotarem, the Gd_2_O_3_@PCD NPs are promising as a targeted CA for early diagnosis of cancer by MRI. Due to the presence of a hydrophobic cavity of CD in the structure of the targeted NPs, these NPs can transport hydrophobic charges, making them cost-effective as potential theranostics agents. Various primary hydroxyl groups at the upper rim and secondary hydroxyl groups at the lower rim of the exterior surface can be selectively modified with a variety of functional moieties to provide tailored functionalities [9].

Meanwhile, to prevent Gd^+3^ ion from leaching the novel synthesized biocompatible targeted CA, Gd_2_O_3_-based PCD, due to its glucose chemical structure and metabolite similarities to CD, provides the ability to distinguish cancerous cells from normal cells. The proof for this can be seen in-vivo MR images in figures 5 and 7, showing the metastatic axillary lymph node and tumor have been visualized with higher and more prolonged enhancement in tumors, with the greatest contrast visible 30 minutes after injection. Also these figures 1,7, and 8 by showing this novel CA would be delivered in a high concentration to lymph nodes, compensating for the low background concentration in the surrounding healthy tissue. Gd_2_O_3_@PCD has been used for interstitial injections due to their properties of truncated cone chemical structure with excellent biocompatibility, whereby the CAs are absorbed and transported from the interstitial tissue into the collector lymphatics.

Finally, we demonstrated that interstitial MR lymphography with Gd_2_O_3_@PCD allowed clear visualization of the SLN in tumoral mice. Meanwhile, mouse lymph nodes are smaller and have some differences from those of humans, so this experiment should also be performed in large animals to reliably detect metastases in lymph nodes and other possible injection sites, including intestinal, subareolar over the primary tumor site, peritumoral, and intratumoral sites, as well.

## 5. Conclusion

The results of a study for the first time showed the novel introduced Gd_2_O_3_@PCD magnetic nanoparticles complexes possessed higher relaxation effectiveness, lower cytotoxicity, and significantly higher enhanced signal intensities of axillary lymph nodes in mice with lower injection doses than that of Dotarem. Gd_2_O_3_@PCD NPs are potentially a passive targeting metabolic CA for metastatic lymph nodes imaging with molecular MRI applicability due to their long-term imaging ability, considerable payload, and accumulative concentration capacity that can be used in future nuclear medicine PET-MRI molecular imaging and lymphography methods.

## Figures and Tables

**Figure 1:** (a, b, c) Schematic representation of the synthesis of the passive targeted Gd-based Nano-CA and Lymph node detection by using an MRI contrast agent that binds to PCDs. Metabolically nanoparticles with a size between 20 and 40 nm have a rapid uptake into metastatic axillary lymph nodes as well as an extremely long retention time.

**Figure 2:** (a) TEM images of Gd_2_O_3_@ PCD NPs, TEM images reveal that Gd_2_O_3_@PCD NPs are spherical and uniform that could be visualized separately with clear grains in nano dimensions with a range of 20–30 nm. (b) Intensity-based DLS data on same 100 *µ*g/ml dispersion of Gd_2_O_3_@PCD (∼45 nm mean size). This result showed that Gd_2_O_3_ nanoparticles had a hydrodynamic diameter distribution of 45 ± 7.6 nm with a PDI of 0.36 that is the proper size. (c) Zeta potential of Gd_2_O_3_@PCD and Gd_2_O_3_NPs. The Zeta potentials value of Gd_2_O_3_ and Gd_2_O_3_@PCD NPs were (+17.5 mv) and (−37.5 mv), respectively, which confirms adequate chemical surface repulsion potential of Gd_2_O_3_ coating with PCD.

**Figure 3:** (a) T_1_−weighted images of Gd2O3@CD NPs and Dotarem at various Gd concentrations.^.^ (b) T_1_−mapping of (a). (c) *R*_1_ (1/T1) diagram of (a), showing *r*_1_ (mM^−1^·s^−1^); the slope of *R*_1_ vs. concentration, as specific relaxivities of 3.98 and 2.71 mM^−1^·s^−1^ for Gd_2_O_3_@CD NPs and Dotarem, respectively, show efficiently shorten T_1_ values of Gd_2_O_3_@PCD NPs leading to significantly increased signal intensity in T_1_W images compared to Dotarem even in low concentrations of Gd_2_O_3_@PCD NPs nanoparticles in MRI.

**Figure 4:** Histopathology of lymph node tissue and tumor mass. (a) Schematic of lymph nodes in mice with 4T_1_ tumor. (b) Red arrows and ROI, respectively, axillary LN. (c and d) Black Arrows: Metastatic tumor cells in axillary LN, H&E stain, Magnification: X100-X400. (e, f, and g) Original tumor mass, Mitotic figures, arrowheads: metastatic cells in the blood and lymphatic vessels. Focal metastasis of breast cancer (arrows) was seen in the harvested lymph node.

**Figure 5:** MR Imaging of tumor in a mouse model with 4T_1_ carcinoma in the right lower limb. Example of white arrows in the muscle of right femur tumor. (a) Schematic of axillary lymph nodes and injection method in mice. (b and c) MR image before and after injection of Gd_2_O_3_@PCD and Dotarem (0.6 mM). Gd_2_O_3_-PCD showed higher and more prolonged enhancement in tumors, with the greatest contrast visible at 15 minutes.

**Figure 6:** Time-intensity curves of the tumor in mice. Gd_2_O_3_-PCD show higher and more prolonged enhancement in tumors, with the greatest contrast visible at 15 minutes. Error bars are standard errors.

**Figure 7:** (a and b) MR Imaging of the lymph node in a mouse model before and after a subcutaneous injection of Gd_2_O_3_@PCD and Dotarem. In a comparison of pre- and post-contrast images, Gd_2_O_3_@PCD and Dotarem are enhanced in LN, whereas Dotarem uptake is confined to all slices. An example of white arrows in the right axillary lymph node and yellow arrows showed the lumbar-aortic lymph node weakly visible in the original coronal image.

**Figure 8:** Time-intensity curves of the two lymph nodes: (a) axillary, (b) (lumbar-aortic) in tumoral mice, Gd_2_O_3_@PCD showed stronger and more prolonged enhancement of lymph nodes than Dotarem. Error bars are standard errors.

## Data Availability

The data used to support the findings of this study are available from the corresponding author upon request.
